RETRACTED

# Anti-Tumor Activity of a Novel Compound-CDF Is Mediated by Regulating miR-21, miR-200, and PTEN in Pancreatic Cancer

**DOI:** 10.1371/journal.pone.0017850

**Published:** 2011-03-09

**Authors:** Bin Bao, Shadan Ali, Dejuan Kong, Sanila H. Sarkar, Zhiwei Wang, Sanjeev Banerjee, Amro Aboukameel, Subhash Padhye, Philip A. Philip, Fazlul H. Sarkar

**Affiliations:** 1 Department of Pathology, Wayne State University, Detroit, Michigan, United States of America; 2 Division of Hematology/Oncology Karmanos Cancer Institute, Wayne State University, Detroit, Michigan, United States of America; 3 Dr. D. Y. Patil University, Pimpri, Pune, India; University of Pennsylvania, United States of America

## Abstract

**Background:**

The existence of cancer stem cells (CSCs) or cancer stem-like cells in a tumor mass is believed to be responsible for tumor recurrence because of their intrinsic and extrinsic drug-resistance characteristics. Therefore, targeted killing of CSCs would be a newer strategy for the prevention of tumor recurrence and/or treatment by overcoming drug-resistance. We have developed a novel synthetic compound-CDF, which showed greater bioavailability in animal tissues such as pancreas, and also induced cell growth inhibition and apoptosis, which was mediated by inactivation of NF-κB, COX-2, and VEGF in pancreatic cancer (PC) cells.

**Methodology/Principal Findings:**

In the current study we showed, for the first time, that CDF could significantly inhibit the sphere-forming ability (pancreatospheres) of PC cells consistent with increased disintegration of pancreatospheres, which was associated with attenuation of CSC markers (CD44 and EpCAM), especially in gemcitabine-resistant (MIAPaCa-2) PC cells containing high proportion of CSCs consistent with increased miR-21 and decreased miR-200. In a xenograft mouse model of human PC, CDF treatment significantly inhibited tumor growth, which was associated with decreased NF-κB DNA binding activity, COX-2, and miR-21 expression, and increased PTEN and miR-200 expression in tumor remnants.

**Conclusions/Significance:**

These results strongly suggest that the anti-tumor activity of CDF is associated with inhibition of CSC function via down-regulation of CSC-associated signaling pathways. Therefore, CDF could be useful for the prevention of tumor recurrence and/or treatment of PC with better treatment outcome in the future.

## Introduction

Pancreatic cancer (PC) is one of the most lethal malignant diseases with worst prognosis, which is ranked as the fourth leading cause of cancer-related deaths in the United States [1]. Over the past two decades, numerous efforts have been made in improving treatment and survival PC patients but the outcome has been disappointing. This disappointing outcome is due to many factors among which *de novo* resistance (intrinsic) and acquired (extrinsic) resistance to conventional therapeutics (chemotherapy and radiation therapy) including gemcitabine alone or in-combination with other cytotoxic or targeted agents. Emerging evidence suggest that the resistance could in fact be due to the enriched existence of tumor initiating cells, also classified as cancer stem-like cells (CSC) in a tumor mass [2]–[6]. The CSCs have the capacity of self-renewal and the potential to regenerate into all types of differentiated cells giving rise to heterogeneous tumor cell populations in a tumor mass, which contributes to tumor aggressiveness [2]–[6]. Thus, the failure to eliminate these special cells is considered to be one of the underlying causes of poor treatment outcome with conventional therapeutics, suggesting that newer and novel therapeutic strategies must be developed for the targeted killing of drug resistant CSCs in order to eradicate the risk of tumor recurrence for improving the survival of patients diagnosed with PC.

RETRACTED

In search of novel yet non-toxic agents, attention has been focused on natural agents for several years. One such agent is curcumin (diferuloylmethane), which is derived from the plant Curcuma longa (Linn) grown in tropical Southeast Asia [7]–[9]. Curcumin has been shown to inhibit the growth of a variety of tumor cells; however, the poor bioavailability of curcumin limits its application in the clinic. Recently, we have developed a novel synthetic analogue of curcumin, 3,4-difluoro-benzo-curcumin [we named it as Difluorinated-Curcumin or in short CDF [10], [11]], which showed greater bioavailability in pancreatic tissues, and also inhibited cell growth, DNA-binding activity of NF-κB, Akt, COX-2, and the production of PGE_2_ and VEGF, and caused induction of miR-200 and inactivation of miR-21 in PC cells [12]. Since miR-200 is associated with the acquisition of epithelial to mesenchymal transition (EMT), which is also believed to be associated with CSCs or cancer stem-like cells, here we investigated the effects of CDF on CSC function.

Here we report, for the first time, that CDF could inactivate many functions of CSCs including self-renewal capacity as demonstrated by the inhibition of sphere-forming (pancreatospheres) ability of drug-resistant PC cells, which was consistent with inactivation of CSC biomarkers such as CD44 and EpCAM. We also showed anti-tumor activity of CDF alone and in-combination with gemcitabine, which was consistent with inactivation of miR-21, and consequently increased expression of PTEN, attenuation of the DNA binding activity of NF-κB inhibition in the expression of COX-2, and activation in the expression of miR-200 in tumor remnants of a xenograft mouse model of human PC, all of which provide convincing *in vivo* activity of CDF which is consistent with *in vitro* findings.

RETRACTED

## Results

AsPc-1 and MIAPaCa-2 cell lines and their clones were chosen for this study because of their relatively resistant nature. The CSC characteristics of these cell lines using stem cell markers' Lin28B and Nanog by RT-PCR, and EpCAM and CD44 by western blot showed an increase in expression level in the PC-GTR cell lines compared to their parental cell lines (Figure 1). Hence we chose these to test our hypothesis that CDF is more effective than curcumin even in resistant cell lines and also their resistant clones–GTR.

**Figure 1:** Comparative expression of Lin28B (A) and Nanog (B) mRNA by qRT-PCR showed increased expression in resistant cell lines compared to parental cell lines, supporting the CSC characteristics of these cell lines. The characteristics of CSCs were further confirmed by the protein expression of EpCAM and CD44 (**C**).

### CDF strongly prevents clonogenicity and invasion of PC cells compared to gemcitabine and curcumin

We selected the concentration of 20 nmol/L of gemcitabine and 4 µmol/L of curcumin or CDF to conduct clonogenic assay following our previous publication [12]. The results demonstrated that there was a significant reduction in clonogenicity of AsPC-1 and MIAPaCa-2 cells treated with curcumin and CDF, but not with gemcitabine (Figure 2A). However, CDF treatment had a much greater and significant reduction in colony formation compared to curcumin. AsPC-1-GTR and MIAPaCa-2-GTR cells had an 80% reduction of clonogenicity with CDF treatment, whereas, only 20–30% reduction of clonogenicity was observed with gemcitabine or curcumin treatment (Figure 2A). Overall, CDF treatment showed a significant reduction in clonogenicity of human PC cells, suggesting the superiority of CDF.

**Figure 2:** CDF and Curcumin decreased clonogenicity and invasion in AsPC-1, AsPC1-GTR, MIAPaCa-2, and MIAPaCa-2-GTR cells. Clonogenic assay (A) Invasion assay (B). Fluorescence of the invaded cells was read using ULTRA Multifunctional microplate reader (TECAN) at excitation/emission wavelengths of 530/590 nm. Basal level of ABCG2 expression showing relatively higher expression in drug resistant cell lines (**C**).

CDF or curcumin treatment decreased PC cell migration and invasion. The results showed that 4 µmol/L of curcumin had minimal inhibition of invasion whereas similar concentration of CDF showed significant inhibition of invasion (Figure 2B). The basal level of ABCG2 expression was found in parental cell lines (*de novo* drug resistant cells); however, the level of expression of ABCG2 was further increased in drug resistant (acquired drug resistant) cell lines (Figure 2C).

RETRACTED

### CDF inhibited viability of human PC cells more than curcumin and gemcitabine as evaluated by MTT assay

Initially MTT assay was conducted to examine the effect of different concentrations of gemcitabine (1 to 50 nmol/L), and curcumin or CDF (2–6 µmol/L) on cell survival after 72h of treatment (data not shown). Subsequently, 4 µmol/L of CDF or curcumin, and 20 nmol/L of gemcitabine were used to treat individually as well as in combination with gemcitabine for 72h. The results showed that CDF treatment in combination with gemcitabine caused a remarkable reduction of cell survival in all four cell lines compared to curcumin and gemcitabine combination treatment (Figure 3). Furthermore, analysis of drug combination treatment showed that the combination index after treatment with CDF in combination with gemcitabine was less than 1.00 (Figure 3), suggesting the synergistic effect of CDF combination. In contrast, the combination index with curcumin and gemcitabine was more than 1.00 (Figure 3), showing non-synergistic effect. Overall, these results suggest that CDF caused a much more significant reduction of cell survival in PC cells, compared to gemcitabine/curcumin alone or their combinations compared to CDF and gemcitabine combination.

**Figure 3:** CDF and its combination with gemcitabine inhibited cell viability. MTT assay was conducted in all four cell lines after 72h of treatment with CDF, curcumin, or its combination with gemcitabine. Untreated control has been assigned a value of 100%. The p value shown represents comparisons between single agent and their combinations by using paired t-test. The combination Index (CI) <1 for CDF and Gemcitabine combination indicates synergism.

### CDF remarkably increased pancreatosphere disintegration of PC cells

To examine the effect of treatments on the sphere forming ability of PC cells (pancreatosphere) and disintegration of pancreatospheres, we conducted sphere disintegration assay for 10 days to generate the formation of pancreatospheres, followed by 5 days of drug treatment. The results show that there was a remarkable increase of sphere disintegration by curcumin and CDF treatment, not by gemcitabine treatment (Figure 4). However, the greatest effect on disintegration was observed in response to the CDF treatment (Figure 4), once again suggesting that CDF is much more superior in inhibiting the functions of cancer stem-like cells.

**Figure 4:** CDF remarkably increased disintegration of pancreatospheres in AsPC-1, AsPC1-GTR, MIAPaCa-2, and MIAPaCa-2-GTR cells. P values were calculated by the paired *t* test.

RETRACTED

### CDF inhibited pancreatospheres formation in PC cells

To examine the effect of drugs on CSC self-renewal capacity in PC cells, we conducted sphere formation assay for 1 week and four weeks (Figure 5A and B). The results indicated that CDF in combination with gemcitabine completely eliminated pancreatospheres formation after four weeks of treatment compared to gemcitabine and curcumin combination in PC cells even in gemcitabine-resistant PC cells, suggesting that CDF may cause the pancreatospheres more sensitive to gemcitabine than that of curcumin treatment, and could be useful for targeted killing of CSCs. Figure 5C shows the effect of different concentration of gemcitabine and CDF on 2^nd^ passage of pancreatospheres in pre-treated primary pancreatospheres of AsPC-1 cells. CDF treatment remarkably inhibited 2^nd^ passage of pancreatospheres in a dose-dependent manner. Furthermore, CDF-pre-treated cells exhibited a greater effect than non-CDF-pre-treated cells.

**Figure 5:** CDF decreased the formation of pancreatospheres in AsPC-1 and AsPC-1-GTR cells 1 week treatment (A); 4 weeks treatment (B); AsPC-1 and CDF-pre-treated AsPC-1 cells treated with gemcitabine and CDF (C). A significant reduction in pancreatospheres was observed in cells treated with CDF shown by asterisk

### CDF decreased CD44 and EpCAM expression in pancreatospheres of PC cells

We examined the effect of drugs on CSC biomarkers, CD44 and EpCAM in pancreatospheres of AsPC-1 and AsPC-1-GTR cells by confocal microscopy (Figure 6). The results indicate that CDF decreased CD44 and EpCAM expression in pancreatospheres, suggesting the inhibitory effect of CDF on pancreatosphere formation may be associated with the inhibition of CD44 and EpCAM expression.

**Figure 6:** CDF treatment decreased the expression of CD44 and EpCAM, the known markers of CSCs. Expression in pancreatospheres of AsPC-1 and AsPC-1-GTR cells was assessed by confocal microscopy (Magnification X250).

### CDF in combination with Gemcitabine inhibited Pancreatic Tumor Growth in vivo much more than curcumin combination

We have used a subcutaneous xenograft tumor model where the tumor was induced by MIAPaCa-2 cells in CB17-SCID mice. CDF treatment in combination with gemcitabine significantly inhibited tumor growth in MIAPaCa-2 tumors much more than curcumin and gemcitabine combination (Figure 7A) as well as compared to either untreated controls or those treated with a single drug. The mice did not show any weight loss during the treatment period (30 days), suggesting that these treatment had no major adverse effects on animals.

RETRACTED

**Figure 7:** CDF exhibited anti-tumor activity in MIAPaCa-2 cells induced tumors in a xenograft mouse model, which was consistent with inhibition of NF-κB DNA binding, COX-2, miR-21, and caused re-expression of miR200 in tumor remnants. Anti-tumor activity and changes in tumor weight from each group of animals (**A**). The arrow indicates starting day of the treatment. NF-κB DNA binding activity of tumor tissues; and NF-κB competition control study with unlabeled NF-κB oligonucleotide (**B**). Western blots analysis of COX-2, PTEN and β-actin expression in tumor remnants (**C**); miR-21, miR-200b and miR-200c expression in tumor remnants as measured by real-time RT-PCR (**D**). P values were calculated by the paired *t* test.

### CDF with Gemcitabine significantly decreased NF-κB Activation *in vivo*

NF-κB activation was determined in the CDF or curcumin, and/or gemcitabine treated tumor remnants derived from MIAPaCa-2 cells induced tumors as shown above. CDF and curcumin as single agent down-regulated NF-κB activation whereas gemcitabine activated NF-κB level, which was abrogated in combination treatment with CDF. The combination treatment of CDF with gemcitabine showed a significant decrease in NF-κB level compared to curcumin and gemcitabine treatment (Figure 7B), suggesting that the inactivation of NF-κB could be one of the molecular mechanisms by which CDF elicits its anti-tumor activity against PC tumors.

### CDF effects on protein expression *in vivo*

The COX-2, PTEN, and β-actin expression was determined by Western blot. A significant down-regulation in the expression of COX-2 was observed in both the combination, but the effect was more pronounced in CDF combination group. The expression of phosphatase and tension homolog (PTEN), a tumor suppressor gene was found to be decreased in MIAPaCa-2 cells; however, the expression of PTEN was up-regulated when treated with CDF (Figure 7C). These results suggest that CDF is much more effective than curcumin. Since PTEN is a known target of miR-21, which has been reported to be up-regulated in PC [13]–[15], we assessed the expression levels of miR-21 in tumor remnants as shown below.

### Modulation in the expression of miR-21 and miR-200 family *in vivo*

We determined the expression levels of miR-21, miR-200b and miR-200c in MIAPaCa-2 tumors by real time RT-PCR. Over-expression of miR-21 was observed in MIAPaCa-2 tumors whereas we found a significant reduction in the expression of miR-21 in tumors treated with either CDF alone or in combination with CDF and gemcitabine (Figure 7D). We further determined the expression levels of miRNA-200b and miR-200c in tumor tissues which are known regulators of EMT and found to be significantly low in MIAPaCa-2 cells (Figure 7D). In contrast, we found that the CDF treatment with or without gemcitabine combination showed increased expression of both miR-200b, and miR-200c, but the effect with curcumin or its combination was minimal, suggesting the superiority of CDF in suppressing the expression of miR-21, resulting in the re-expression of PTEN, and re-expression of miR-200 which could be responsible for the reversal of EMT phenotype in cells treated with CDF. Overall, these results suggest that the phenotypic characteristics of MIAPaCa-2 tumors are consistent with enriched population of CSCs and EMT characteristics, and these drug resistant cells could be killed either by CDF alone or in combination with gemcitabine.

RETRACTED

### Pancreatospheres enhanced tumor growth *in vivo*

Under traditional experimental conditions, we normally inject one million cells for assessing tumor growth; however, for investigating the greater potential of tumor growth by pancreatospheres, we injected only 5,000 cells in mice as a proof-of-concept study. The tumor weight was remarkably increased as the days progressed (Figure 8A). The level of miR-21 was increased between tumors implanted with one million of parental cells compared to pancreatospheres (Figure 8B). The animal was euthanized after 30 days because of tumor burden, and gross tumors are shown in Figure 8C indicating larger tumors as well as loco-regional lymph node metastasis whereas tumors derived from parental cells did not show any metastasis over a period of 30 days. The tumor-derived cells showed significant inhibition of pancreatospheres when treated with CDF (Figure 8D). Overall, these results suggest that CSCs (pancreatospheres) can be grown in mice and CDF could be useful for the killing of these drug resistant cells (Figure. 8).

**Figure 8:** Tumor growth pattern of pancreatospheres derived from MIAPaCa-2 cells. (**A**). 5,000 pancreatospheres were inoculated in mice using 1∶1 matrigel, progressive tumor growth over a period of 30 days. Moderate increase in the expression of miR-21 as measured by real-time RT-PCR was observed in tumors derived from pancreatospheres compared to tumors derived from parental cells by injecting one million cells and tumor was assessed over the same period of time (**B**). Photographs showing tumor growth, arrow points to tumor and asterisk (*) refers to loco-regional lymph node metastasis whereas we did not find any metastasis when one million parental cells were injected (**C**). Tumor cells harvested from the tumors derived from pancreatospheres were treated with CDF showed significant inhibition in the formation of pancreatospheres (**D**).

RETRACTED

## Discussion

In this study, we have demonstrated that a synthetic analogue of curcumin, CDF, is significantly more effective compared to curcumin in the killing of gemcitabine-resistant pancreatic cancer (PC) cells that consists high proportion of cells with cancer stem cells (CSCs) or cancer stem-like cells characteristics. The inhibition of cell growth could in part be due to better cellular uptake, retention and reduced metabolic inactivation of CDF by PC cells, which is consistent with our published findings on cellular and animal pharmacokinetics data [10], [11]. Our previous reports indicate that CDF inhibits NF-κB and COX-2 activity in PC cells *in vitro* [12]. Here we confirm these observations *in vivo* using a mouse xenograft model. Thus, the killing of gemcitabine-resistant PC cells by CDF is associated with inactivation of NF-κB and COX-2 signaling pathway which is very important because these pathways are known to contributes to drug-resistance of PC cells to chemotherapeutic agents [16]–[18].

CSCs comprises only a very small proportion of cells in a tumor mass and posses the ability to self-renew and give rise to differentiated tumor cells [3]–[5], [19]. The CSC theory has fundamental clinical implications especially because CSC has been identified in many malignant tumor tissues including pancreatic cancers and considered to be highly resistant to chemo-radiation therapy than differentiated daughter cells [3]–[5], [20]; however, CSCs isolated from human tumors are usually insufficient for further mechanistic studies. The existence of CSCs provides an explanation for the clinical observation that tumor regression alone may not correlate with patient survival [21] because of tumor recurrence, which is in part due to the presence of CSCs. Therefore, targeting self-renewal pathways and the killing of CSCs might provide more specific approach for eliminating cells that are the root cause of tumor recurrence. A potential challenge in this regard is the development of therapies that selectively affect CSCs while sparing normal stem cells that may rely on similar mechanisms for self-renewal. In this study, we have demonstrated that CDF not only inhibit cell growth of PC cells, but also inhibit CSC self-renewal capacity as assessed by sphere formation (pancreatospheres) assays. Therefore, CDF could have a greater potential to inhibit cancer growth as documented by our xenograft mouse model of gemcitabine resistant PC cells, which appears to be mediated via inhibition of CSC self-renewal capacity.

Emerging evidence suggests the role of microRNA (miRNA) in many biological processes [22]–[25]. Among many miRNAs, miR-21, commonly considered as an oncogene, is over-expressed in many solid tumors including PC and has been reported to be associated with tumor progression, poor survival and drug resistance [13], [14], [26], [27]. In our previous report, we have demonstrated that the expression of miR-21 is up-regulated in gemcitabine-resistant PC cells and that its expression can be significantly down-regulated by CDF treatment *in vitro* [12]. The increased expression of miR-21 is known to be associated with inactivation of PTEN, a know tumor suppressor gene, resulting in activation of PI3K/Akt/mTOR signaling pathway, leading to aggressive tumor growth [15], [28]. In this study, we confirmed that CDF treatment could results in the down-regulation of miR-21, resulting in the up-regulation of PTEN *in vivo*, suggesting that the anti-tumor activity of CDF is associated with up-regulation of PTEN resulting from the inactivation of miR-21 expression.

RETRACTED

In contrast to miR-21, miR-200 family is known as tumor suppressor and they are usually down-regulated in some tumors including PC and the loss of expression of miR-200 family contribute to the acquisition of EMT phenotype and drug resistance. Down-regulation of miR-200 by siRNA technique has been shown to be associated with EMT phenotype while re-expression of miR-200 can result in the reversal of EMT phenotype [29], [30]. In our previous publication [12], we demonstrated that CDF treatment could re-express miR-200 in PC cells. Here we showed, for the first time, that CDF can up-regulate miR-200b and miR-200c in tumor remnants *in vivo*, consistent with significantly greater inhibition of tumor growth in the xenograft mouse model when CDF was used in combination with gemcitabine. These results suggest that the anti-tumor activity of CDF is mediated via re-expression of miR-200 which may potentially results in the reversal of EMT phenotype and could also lead to overcome drug resistance in PC.

In conclusion, CDF showed much more pronounced growth inhibitory effect, inhibited CSC self-renewal consistent with inactivation of CSC biomarkers (CD44 and EpCAM) in PC cells especially in gemcitabine-resistant PC cells compared to curcumin. In xenograft mouse model of human PC tumors induced by MIAPaCa-2 cells, CDF exhibits anti-tumor activity by regulating COX-2, PTEN, miR-21, miR-200, and NF-κB *in vivo*. These results strongly suggest that CDF could be a novel agent for the treatment of PC in general but gemcitabine-resistant PC in particular by attenuating the behavior of CSCs.

## Materials and Methods

### Ethics Statement

This study was carried out in strict accordance with the recommendations in the Guide for the Care and Use of Laboratory Animals of the National Institutes of Health. Any animal found unhealthy or sick were promptly euthanized. The protocol was approved by the Committee on the Ethics of Animal Experiments of Wayne State University institutional Users Animal Care Committee (Permit Number: A-10-03-08).

RETRACTED

### Cell Culture, Drugs and Reagents

Human pancreatic cancer cell lines AsPC-1, and MIAPaCa-2 were purchased from ATCC (Manassas, VA). These two cell lines AsPC-1 and MIAPaCa-2 were exposed to 200 nmol/L of gemcitabine and 5 µmol/L of tarceva (erlotinib) every other week for about 6 months to create gemcitabine and tarceva resistant (GTR) cell lines, named as AsPC-1-GTR and MIAPaCa-2-GTR, respectively. As a result, AsPC-1, AsPC-1-GTR, MIAPaCa-2, and MIAPaCa-2-GTR were chosen for this study based on their differential sensitivities to gemcitabine. All the cell lines have been authenticated (Applied Genomics Technology Center at Wayne State University) on March 13, 2009 and these authenticated cells were frozen for subsequent use. The method used for testing was short tandem repeat profiling using the PowerPlex 16 System from Promega. Gemcitabine and curcumin were purchased from Eli Lilly (Indianapolis, IN) and Sigma-Aldrich (St. Louis, MO), respectively. CDF was synthesized as described in our earlier publication [10], [11]. Gemcitabine was dissolved in water, whereas CDF and curcumin were dissolved in DMSO with a final concentration of 0.1% DMSO in medium.

### Antibodies

Antibodies against ABCG2, and PTEN were purchased from Santa Cruz (Santa Cruz, CA). Antibody to COX-2 and β-actin was acquired from Cayman Chemicals (Ann Arbor, MI), and Sigma Chemicals (St. Louis, MO).

### Clonogenic assay

Clonogenic assay was conducted to examine the effect of drugs on cell growth in PC cells, as described previously [12]. 5×10^4^ cells were plated in a six-well plate. After 72h of exposure to 20 nmol/L of gemcitabine, 4 µmol/L of CDF or curcumin, the cells were trypsinized, and 1,000 single viable cells were plated in 100-mm Petri dishes. The cells were then incubated for 10 to 12 days at 37°C in a 5% CO_2_/5% O_2_/90% N_2_ incubator. Colonies were stained with 2% crystal violet and counted.

### Invasion assay

The invasive activity of cells was tested by using BD BioCoat Tumor Invasion Assay System (BD Biosciences, Bedford, MA) according to the manufacturer's protocol as described previously [31]. Briefly 5×10^4^ cells were seeded with serum free medium supplemented with curcumin or CDF into the upper chamber and bottom wells were filled with complete medium in the system. The, fluorescence was read using Microplate Reader (TECAN) at 530/590 nm and were photographed.

RETRACTED

### Cell survival assay

MTT assay was conducted using AsPC-1, AsPC-1-GTR, MIAPaCa-2, and MIAPaCa-2-GTR as described previously [12] after 72 h of treatment. Combination index and Isobologram for combination treatment were also calculated and plotted using CalcuSyn software (Biosoft, Cambridge, United Kingdom) to determine synergy based on the method of Chou and Talalay [32].

### Sphere formation/disintegration assay

Single cell suspensions of cells were plated on ultra low adherent wells of 6-well plate at 1,000 cells/well in sphere formation medium [33]. After 7 days, the spheres termed as “pancreatospheres” were collected by centrifugation and counted [33]. For sphere disintegration assay, 1,000 cells/well were incubated for 10 days, following 5 days of drug treatment, which examined the effect of drug treatment on disintegration of pancreatospheres as described previously [33]. The pancreatospheres were collected by centrifugation and counted under a microscope.

### Confocal microscopy

Single cell suspensions of AsPC-1 and AsPC-1-GTR cells were plated using ultra low adherent wells of 6-well plate at 3,000 cells/well in sphere formation medium. After 7 days of treatment, the pancreatospheres were collected by centrifugation, washed with 1xPBS, and fixed with 3.7% parformaldehyde. CD44 and EpCAM antibodies were used for immunostaining assay, as described previously [29]. The CD44 or EpCAM-labeled pancreatospheres were photographed by confocal microscopy (Leica TCS SP5) using software LAS AF 1.2.0 Build 4316.

### Protein extraction and Western blot analysis

Proteins were extracted from all four cell lines and also from animal tumor tissues as described previously [12]. Relative level of ABCG2 was evaluated for all four cell lines. The effects on COX-2, PTEN and β-actin expression were evaluated on tumor tissues by Western blot analysis. as described previously [12].

### Animal Experiments

The animal protocol was approved by the Animal Investigation Committee, Wayne State University, Detroit, MI. Female CB17 SCID mice 4 wks old were purchased from Taconic Farms (Germantown, NY) and fed Lab Diet 5021 (Purina Mills, Inc., Richmond, IN). Small fragments of the MIAPaCa-2 xenograft were implanted subcutaneously and bilaterally into mice for the drug-efficacy trials. Once the mice developed palpable tumors, they were randomly selected into the following treatment groups (n  =  5/group): (1) untreated control; (2) CDF (5 mg/mouse/day), intragastric once daily for 12 days; (3) curcumin (5 mg/mouse/day), intragastric once daily for 12 days; (4) gemcitabine (1 mg/mouse/day), intravenous every third day for a total of three doses; (5) CDF and gemcitabine using the doses indicated above; (6) curcumin and gemcitabine using the doses as indicated above. Tumor measurements and changes in weight were performed and tissue was stored at −70°C for RNA and protein extraction.

RETRACTED

### Electrophoretic Mobility Shift Assay (EMSA) assay for assessing the DNA binding activity of NF- κB

Nuclear proteins were prepared from tumors tissue using a Dounce homogenizer with 400 µl of ice cold lysis buffer extracted as described earlier [34]. EMSA was performed using the Odyssey Infrared Imaging System with NF-κB IRDye labeled oligonucleotide from LI-COR, Inc. (Lincoln, NE). Ten µg of the nuclear protein extract was used as described earlier [34]. The NF-κB competition control study was conducted using unlabeled NF-κB consensus oligonucleotide. The samples were loaded and run at 30 mA for 1 hour. The gel was scanned using Odyssey Infrared Imaging System (LI-COR, Inc.).

### TaqMan miRNA Real-Time Reverse Transcriptase-Polymerase Chain Reaction (RT-PCR)

To determine the expression of miRNAs (miRNA-200b, miR-200c, and miR-21) in MIAPaCa-2 tumors, we used TaqMan MicroRNA Assay kit (Applied Biosystems) following manufacturer's protocol. 5 ng of total RNA was reverse transcribed and real-time PCR reactions were carried as described earlier [30], using Smart Cycler II (Cepheid). Data were analyzed using C_t_ method and were normalized by RNU6B expression.

### Growth of CSC in xenograft model

5,000 pancreatospheres were isolated and implanted in mice with 1:1 matrigel. The growth rate was observed for a period of 30 days. RNA was extracted from the tumor tissue for subsequent molecular assays as presented under figure legend.

### Statistical Analysis

Comparisons of treatment outcome were tested for statistical difference by the paired *t* tests. Statistical significance was assumed at a *P* value of <0.05.
